This article has been retracted.

# Effects of Different Ovulation Induction Regimens on Sex Hormone Levels and Serum CTRP3 and CTRP15 Levels in Patients with Polycystic Ovary Syndrome (PCOS)

**DOI:** 10.1155/2022/6027878

**Published:** 2022-04-12

**Authors:** Maohua Ren, Jianrong Liu, Yanling Zhang, Linxiao Fan

**Affiliations:** ^1^The Fifth Clinical Medical College of Shanxi Medical University (Shanxi Provincial People's Hospital) Gynaecology and Obstetrics 030012, China; ^2^The Fifth Clinical Medical College of Shanxi Medical University (Shanxi Provincial People's Hospital) Department of Reproductive Medicine 030012, China

## Abstract

**Objective:**

A retrospective cohort study aimed to explore the effects of different ovulation induction regimens on the levels of sex hormones and serum C1q/TNF-related protein-3 (CTRP3) and C1q/TNF-related protein-15 (CTRP15) in patients with PCOS.

**Methods:**

A total of 100 patients with PCOS treated in the department of gynecology and obstetrics from February 2019 to April 2021 in our hospital were enrolled. The patients were arbitrarily assigned into control group and study group. The treatment effect, pregnancy rate, ovulation rate, follicle size, thickness of endometrium, number of mature follicles and ovulation, serum levels of follicle stimulating hormone (FSH), luteinizing hormone (LH), estradiol (E2), testosterone (T), serum CTRP3, CTRP15 and menstrual score were compared.

**Results:**

There exhibited no statistical difference in baseline clinical data between the two kinds of patients. The therapeutic effects were compared, the effective rate was 98.00% in the study group, 13 cases in the control group, 20 cases in the effective group and 7 cases in the control group, and the effective rate was 86.00%. The effective rate in the study group was higher (P <0.05). The size of follicles and the thickness of endometrium in the two groups were compared before and after intervention. There exhibited no significant difference in the size of follicles and the thickness of endometrium before and after intervention (P >0.05). The size of follicles and the thickness of endometrium in the study group were significantly higher (P <0.05). The size of follicles and the thickness of endometrium in the study group were significantly higher (P <0.05). There exhibited no significant difference in the number of mature follicles and ovulation before and after intervention (P >0.05). After intervention, the number of mature follicles and ovulation in the two groups increased. The number of mature follicles and ovulation in the study group were (4.76 ± 0.90) and (4.48 ± 0.73), respectively, which were higher compared to the control group (2.45 ± 0.86) and (2.82 ± 0.84), respectively (P <0.05). The levels of serum LH, FSH, E2 and T were not significantly different before and after intervention. After the intervention of different ways of ovulation induction, the levels of serum LH, FSH, E2 and T in the two groups continued to decrease, and the levels of the above sex hormones in the study group were significantly lower (P <0.05). The menstrual score and the levels of serum CTRP3 and CTRP15 were compared before and after intervention. After intervention, the menstrual score of patients in both groups decreased, and the menstrual score of the study group was lower. In addition, the levels of serum CTRP3 and CTRP15 in the two groups decreased after intervention. Compared with the control group, the levels of CTRP3 and CTRP15 in the study group were lower after intervention (P <0.05). The ovulation rate and pregnancy rate of the two groups were compared. In the study group, there were 45 ovulation cases, the ovulation rate was 90.00% (45/50), the pregnancy rate was 33 cases, the pregnancy rate was 66.00% (33/50), and the ovulation rate in the control group was 31 cases, the ovulation rate was 62.00% (31/50), the pregnancy rate was 20 cases, and the pregnancy rate was 40.00% (20/50). The ovulation rate and pregnancy rate in the study group were higher (P <0.05).

**Conclusion:**

Different ovulation induction regimens have different effects on the levels of sex hormones and serum CTRP3 and CTRP15 in patients with PCOS. Long-acting follicular phase regimens can effectively promote the therapeutic effect of patients and increase the ovulation rate and pregnancy rate. In addition, it can also reduce the levels of serum LH, follicle stimulating FSH, E2 and testosterone T, and help to promote the levels of serum CTRP3 and CTRP15, which is worth popularizing and applying in clinic.

## 1. Introduction

PCOS is a complex and heterogeneous endocrine disease, which is characterized by hyperandrogenemia, oligoovulation and metabolic abnormalities in clinic or laboratory, such as insulin resistance, overweight or obesity, type II diabetes, abnormal blood lipid metabolism and cardiovascular system, which have a far-reaching impact on patients' quality of life, fertility and long-term health [1, 2]. An epidemiological study in China found that the incidence of PCOS is about 5.6%, which is the most common disease that causes ovulation disorders in women of childbearing age. The prevalence rate of foreign women in the same period is about 6% 15% [3]. So far, the exact cause of PCOS is still unclear, and it is considered to be affected by many complex factors such as heredity and environment [4–6]. Studies have indicated that the incidence of PCOS has a certain degree of correlation with families. Genome-wide association analysis (GWAS) of relatives of PCOS has proved that there are multiple genes and multiple gene loci associated with the pathogenesis of PCOS [7–10]. In addition, different personality, psychological and emotional state, nutritional status, lifestyle and intestinal microflora disorder and other factors are also considered to be closely related to the pathogenesis of PCOS [11]. Some scholars have scored the psychological and emotional health status of women with PCOS and women without PCOS and found that the scores of patients are lower than those of normal people, indicating that PCOS is also affected by bad emotions and psychology [12–15]. The pathophysiological abnormalities of PCOS include the disorders of glucose, protein, lipid metabolism, neurohumoral regulation and ovarian regulation, which will have adverse effects on the endocrine and reproductive function of patients [16]. If not timely treatment of its long-term complications such as diabetes, cardiovascular disease, endometrial cancer, hypertension will also affect life and health [17].

PCOS emphasizes the principle of individualized treatment: for women without fertility requirements, it is mainly to reduce androgen, adjust menstrual cycle, and prevent complications; for women with fertility needs, increase the induction of ovulation and promote fertility treatment [18]. Patients with PCOS often have infertility induced by ovulation disorders and need to be assisted by in vitro fertilization (IVF). At present, the commonly employed COS regimens include long-term follicular phase regimen, long-term antagonist regimen, but there is no unified standard for COS regimen in patients with PCOS [19]. Some studies suggest that gonadotropin-releasing hormone agonist (GnRH-a) is employed to down-regulate the pituitary gland in the long-term follicular phase regimen. It can reduce the secretion of luteinizing hormone (LH) and promote the disorder of endocrine and metabolism in patients with PCOS. Theoretically, it may reduce the adverse effects of high androgen and high LH on follicular development and subsequent pregnancy, and obtain a better pregnancy outcome [20]. Drug therapy is still employed as a first-line treatment for PCOS, but because of the complex etiology and diverse clinical phenotypes of PCOS, it is often unable to achieve high curative effect in a short time, with a long treatment cycle and high recurrence rate. Patients often need to use drugs to control their symptoms for a long time [21]. Clinical experience suggests that only one kind of western medicine or only one kind of traditional Chinese medicine cannot achieve satisfactory therapeutic effect. In this study, 100 patients with PCOS were treated in the department of gynecology and obstetrics in our hospital from February 2019 to April 2021. The research process and results are reported as follows.

## 2. Patients and Methods

### 2.1. General Information

A total of 100 patients with PCOS were treated in the department of gynecology and obstetrics from February 2019 to April 2021 in our hospital. The patients were arbitrarily assigned into control group and study group. In the control group, the age was 21-38 years old, with an average of (27.41 ± 3.63) years, and in the study group, the age was 22-37 years old, with an average age of (27.50 ± 3.58) years. There was no statistical significance in the general data of the two groups. This study was permitted by the Medical Ethics Association, and all patients noticed informed consent.

Inclusion criteria: 1) women of childbearing age who are not pregnant have regular menstruation (the cycle is 27-32 days); 2) patients have good communication skills and no language barrier, and can actively cooperate with relevant scores, examinations and inquiries; 3) gynecological ultrasound does not indicate polycystic changes of the ovary.

Exclusion criteria: 1) patients with severe heart, liver, renal insufficiency, malignant tumors, etc.; 2) patients with long-term or recent infections that have not been cured after treatment, or those whose infection has been cured for less than one year; 3) use of drugs that affect glucose and lipid metabolism and sex hormones in the past 3 months; 4) patients with breast hyperplasia or breast cancer; 5) patients with hypertension; 6) diabetes with vascular involvement. 7) patients with cardio-cerebrovascular diseases; 8) obesity; 9) smokers; 10) poor treatment compliance or incomplete clinical data.

### 2.2. Treatment Methods

The control group was treated with antagonist: from the second to the third day of menstruation, gonadotropin (Gn) was employed according to the patient's age, basal antral follicles, basal follicle stimulating hormone (FSH), Anti-Muller's tube hormone (AMH) and body mass index (BMI). The initial dose was generally 150-300 IU/d. The development of follicles was monitored by ultrasound 4-5 days after ovulation induction, and the levels of sex hormones were measured at the same time, and then every 2-3 days and 24 hours before ovulation. When the diameter of dominant follicle reached 14 mm or LH ≥5mIU/ml, GnRH-ant0.125-0.25 mg/d was added to the day of HCG injection. Trigger HCG6000-10000 IU or Ezer 250ug when the maximum follicle diameter ≥18 mm or at least 3 follicles ≥17 mm. 37 hours after the trigger, the eggs were extracted by transvaginal ultrasound. Embryo culture was carried out in accordance with the standard operation of the embryo laboratory of the center. Embryo transfer was carried out under ultrasound guidance on the third day after egg collection. In order to prevent the occurrence of OHSS, fresh cycle embryo transfer may be cancelled when more than 20 eggs were obtained, and all embryos may be vitrified for cryopreservation. After egg extraction, vaginal progesterone gel, injection progesterone or oral progesterone were employed to give luteal support. If the corpus luteum support of pregnancy lasts until 12 weeks of pregnancy, the dosage can be reduced appropriately in accordance with the condition of patient, and the pregnancy outcome can be followed up. The study group adopted the scheme of long-acting follicular phase: long-acting down-regulation of GnRH-a3.75mg was employed in the 2nd-3rd day of menstruation, transvaginal ultrasound and sex hormone levels were measured on the 2nd-35th day of menstruation (FSH<5 U, LH<5 U, LH<5 U, E _ 2 <50 pmol/L, thickness of endometrium <5 mm, diameter of follicles<5 mm). Gn was employed to induce ovulation after complete downregulation. The starting dose of Gn was evaluated according to the patient's age, the number of basic antral follicles, basic FSH, AMH and body mass index, closely monitored follicular development and serum hormone levels, and adjusted the dosage of Gn according to ovarian response.

### 2.3. Observation Index

#### 2.3.1. Therapeutic Effect

Efficacy criteria: effective: clinical symptoms basically disappeared, menstruation basically returned to normal, estrogen level returned to normal range; effective: clinical symptoms were greatly promoted, menstruation was greatly promoted, estrogen level was greatly promoted, but did not return to normal range; ineffective: clinical symptoms did not promote or even worsened, menstruation and estrogen level basically did not promote.

#### 2.3.2. Comparison of Ovulation before and after Intervention

The size of follicles, the thickness of endometrium, the number of mature follicles and ovulation, ovulation rate and pregnancy rate were recorded in the two groups.

#### 2.3.3. Menstrual Scale Score

Using MDQ menstrual symptom scale score, the lower the score, the lighter the symptoms.

#### 2.3.4. Serological Index Collection

All the subjects had an empty stomach for 8 hours and 12 hours, and the blood of the elbow vein was collected on an empty stomach in the morning of the next day. Blood samples were collected from patients with irregular menstruation and amenorrhea on the 3rd to 5th day of menstruation in the control group and PCOS patients with regular menstruation. The following indexes were measured: serum FSH, LH, E2 and T were examined by automatic biochemical analyzer (Roche; model: Cobas6000). Another part of the whole blood sample was kept for 1 hour, then centrifuged with 3000 r/min for 15 minutes and the serum was separated. The serum was sub-packed and stored in the refrigerator at-80°C for the determination of C1q/TNF-related protein-3(CTRP3) and C1q/TNF-related protein-15 (CTRP15).

### 2.4. Statistical Analysis

The data of this experimental study were processed and analyzed by SPSS20.0 software. The measurement data were depicted by (mean + standard deviation). The data between and within groups were compared by t-test, and the percentage was described by percentage (%). The comparison of counting data was analyzed by x2 test, p <0.05.

## 3. Results

### 3.1. Comparison of Therapeutic Effects

We compared the therapeutic effects: 29 cases of markedly effective, 20 cases of effective and 1 case of ineffective in the study group, with an effective rate of 98.00%; in the control group, 13 cases were markedly effective, 20 cases were effective, and 7 cases were ineffective, and the effective rate was 86.00%. Of note, the effective rate of the study group was higher compared to the control group (*χ* 2 = 4.535 P <0.05). All the data results are indicated in Figure 1.

### 3.2. Comparison of Follicular Size and Endometrial Thickness before and after Intervention

We compared the size of follicles and the thickness of endometrium before and after intervention. Before intervention, with no significant difference in the size of follicles and thickness of endometrium (P >0.05). The size of follicles and the thickness of endometrium in the two groups increased, and the size of follicles and the thickness of endometrium in the study group were significantly higher (P <0.05). All the data results are indicated in Table 1.

### 3.3. Comparison of Ovulation before and after Intervention

We compared the ovulation before and after intervention. Before intervention, there exhibited no significant difference in the number of mature follicles and ovulation (P >0.05). The number of mature follicles and ovulation in the study group were significantly higher (P <0.05). The number of mature follicles and the number of ovulation in the study group were significantly higher (P <0.05). All the data results are indicated in Table 2.

### 3.4. Comparison of Sex Hormone Levels before and after Intervention

The levels of serum LH, FSH, E2 and T were not significantly different before and after intervention. After the intervention of different ways of ovulation induction, the levels of serum LH, FSH, E2 and T in the two groups decreased continuously, and the levels of the above sex hormones in the study group were significantly lower (P <0.05). All the data are indicated in Table 3.

### 3.5. 2.5 Comparison of Menstrual Score and Serum CTRP3 and CTRP15 Levels before and after Intervention

We compared the menstrual score and the levels of serum CTRP3 and CTRP15 before and after intervention. After intervention, the menstrual score of the two groups decreased, next, the score of the study group was lower. In addition, the levels of serum CTRP3 and CTRP15 in the two groups decreased after intervention. Of note, the levels of CTRP3 and CTRP15 in the study group were lower after intervention (P <0.05). All the data are indicated in Table 4.

### 3.6. Comparison of Ovulation Rate and Pregnancy Rate

We compared the ovulation rate and pregnancy rate. In the study group, there were 45 ovulation cases, the ovulation rate was 90.00% (45/50), the pregnancy rate was 33 cases, the pregnancy rate was 66.00% (33/50), and in the control group, the ovulation rate was 62.00%. The ovulation rate was 62.00% (31/50), the number of pregnancies was 20 cases, and the pregnancy rate was 40.000% (20/50). The ovulation rate and pregnancy rate in the study group were higher compared to the control group, and the difference was statistically significant (*χ* 2 = 10.746, 4.842, P <0.05). All the data results are indicated in Figure 2.

## 4. Discussion

PCOS is a comprehensive endocrine disorder characterized by persistent anovulation, androgen excess and IR [21]. Its etiology is complex and has not been clarified so far. The clinical manifestations were ovarian polycystic changes, elevated LH/FSH ratio, obesity, acne, hirsutism, menstrual disorders, infertility and so on [5]. Infertility is a common and painful disease in PCOS patients of childbearing age, and its incidence is gradually increasing [22]. According to the diagnostic criteria of Rotterdam PCOS in 2013, the current incidence of PCOS among women of childbearing age in China is 5.6%, while infertility induced by PCOS accounts for 50% to 70% of the total anovulatory infertility, and PCOS patients with assisted reproductive technology towels account for about 50% [23]. The fertility problem has deeply perplexed every patient with infertility due to PCOS, seriously affecting their physical and mental health and family stability, so solving the fertility problem of PCOS patients of childbearing age is a top priority, which should attract the attention of every gynecologist [24]. Epidemiological studies have found that the incidence of PCOS is high in patients with excessive androgen. Another multicenter study found that postmenopausal serum androgen levels in PCOS women with elevated androgen levels were still significantly higher compared to normal people [22]. At present, it is generally believed that hyperandrogenemia is the key factor for a series of abnormal endocrine and metabolic manifestations in patients with PCOS. This study attempts to find a suitable ovulation induction scheme for PCOS patients, on the premise of ensuring the safety of the COS process, to seek an ovulation induction regimen that can obtain a better pregnancy outcome.

During pregnancy, due to the existence of a series of endocrine and metabolic disorders such as hyperandrogenism, insulin resistance and lipid metabolism disorders in patients with PCOS, it has adverse effects on embryonic development and promotes the adverse pregnancy outcome [25]. Therefore, it is of great significance to strengthen the therapeutic effect, ovulation rate and pregnancy rate by means of ovulation induction. The results of this study demonstrated that 29 cases were significantly effective, 20 cases were effective and 1 case was ineffective in the study group, with an effective rate of 98.00%, while in the control group, 13 cases were markedly effective, 20 cases were effective, and 7 cases were ineffective, with an effective rate of 86.00%. The effective rate of the study group was higher. In the study group, there were 45 cases of ovulation, the ovulation rate was 90.000% (45/50), the pregnancy rate was 33 cases, the pregnancy rate was 66.00% (33/50), while in the control group, the ovulation rate was 62.00% (31/50), the pregnancy rate was 20 cases, the pregnancy rate was 40.00% (20/50). The ovulation rate and pregnancy rate in the study group were higher compared to the control group. In addition, related studies have indicated that, the abnormality of follicular size and endometrial thickness can be employed as an option to judge the severity of PCOS [26–28]. It is of great significance to increase the size of follicles and the thickness of endometrium through corresponding treatment. There exhibited no significant difference in follicle size and endometrial thickness before and after intervention (P >0.05). After intervention, the size of follicles and the thickness of endometrium in the two groups increased. The size of follicles and the thickness of endometrium in the study group were (1.51 ± 0.23) and (0.99 ± 0.23), respectively, which were significantly (1.34 ± 0.28) and (0.88 ± 0.20), respectively (P <0.05). The analysis shows that due to the influence of sex hormones and metabolic factors, the patients with PCOS have follicular agenesis, unruptured follicles, decreased oocyte quality, pathological thickening of endometrium and so on. This leads to a significant decrease in the pregnancy rate of the patients. Therefore, in the treatment of ovulation induction, more attention should be paid to the combination of safety and effectiveness of the treatment, and to promote the ovulation rate. A good method of ovulation induction can not only effectively promote the pregnancy rate, but also increase the ovulation rate.

CTRP3 and CTRP15 belong to the CTRP family and share the same globular domain as Adiponectin (APN) [29]. It has been found that APN not only participates in the metabolism of IR and glucose and lipids, but also is closely related to the development of PCOS. Insulin resistance is considered to be the initial link in the occurrence and development of PCOS, but there are few reports on the serum expression and clinical significance of CTRP3 and CTRP15 in infertile patients with PCOS. CTRP3 has been proved to have multiple effects on metabolic diseases. Studies have indicated that its serum level is decreased in patients with obesity and type 2 diabetes, and it is also considered as an anti-inflammatory cytokine, which can promote IR by reducing inflammatory response and regulating insulin signal transduction [29]. A recent study demonstrated that serum CTRP3 levels decreased in infertile women with PCOS [30]. According to this study, there exhibited no significant difference in the number of mature follicles and ovulation before and after intervention. After intervention, the number of mature follicles and ovulation in the two groups increased. The number of mature follicles and ovulation in the study group were (4.76 ± 0.90) and (4.48 ± 0.73), respectively, which were higher compared to the control group (2.45 ± 0.86) and (2.82 ± 0.84), respectively. Next, the menstrual score and the levels of serum CTRP3 and CTRP15 were compared before and after intervention. After intervention, the menstrual score decreased, and then the score of the study group was lower. In addition, the serum levels of CTRP3 and CTRP15 decreased after intervention. The levels of CTRP3 and CTRP15 in the study group were lower after intervention. The levels of CTRP3 and CTRP15 in the study group were significantly lower (11.42 ± 2.27,9.12 ± 1.85 nmol/L). After complete down-regulation of pituitary gland, the hormone level of patients was relatively low, which reduced the adverse effects of long-term high LH and high E2 on endometrium, promoted endometrial receptivity and promoted the result of embryo implantation. In this study, the levels of serum LH, FSH, T and E2 were compared before and after intervention. The levels of serum LH, FSH, T and E2 in the two groups decreased continuously after intervention, and the levels of these sex hormones in the study group were (6.13 ± 1.18) IU/L, (3.78 ± 1.06) IU/L, (1.95 ± 0.63) nmol/L and (103.47 ± 12.08) pg/ml, respectively. All of them were lower than those of the control group (8.92 ± 2.33,5.47 ± 1.35,3.16 ± 0.91,3.16 ± 0.91) IU/L and (119.33 ± 11.24) pg/ml, respectively (P <0.05). The analysis demonstrated that compared with the antagonist regimen, the long-acting GnRH agonist was employed to down-regulate the pituitary gland fully, and the decrease of FSH, LH and E led to the need of a larger dose of Gn stimulation during ovulation induction. Meanwhile, compared with the antagonist group, the antagonist group had no inhibition on follicular development, avoided the stimulation of the ovary by Gn in the early follicular phase, and greatly reduced the days of Gn use. It reduces the time cost and economic cost of patients, and reduces the incidence of OHSS in the process of ovulation induction. Concomitantly, the use of GnRH agonists in follicular phase long-acting long-term plan group and long-term plan group can effectively promote the degree of reproductive endocrine disorder in patients with PCOS, reduce the adverse effects of excessive androgen and LH state on follicular development, coupled with the increase of Gn dose, so a better number of eggs can be obtained, and there are obvious advantages in embryonic development [31–33].

In conclusion, different ovulation induction regimens have different effects on the levels of sex hormones and serum CTRP3 and CTRP15 in patients with PCOS. Long-acting follicular phase regimens can effectively facilitate the therapeutic effect of patients and increase the rate of ovulation rate and pregnancy. In addition, it can also reduce the levels of serum LH, follicle stimulating FSH, E2 and testosterone T, and help to promote the levels of serum CTRP3 and CTRP15, which is worth popularizing and applying in clinic. However, the sample size of this study is limited, and our conclusions and molecular mechanisms need to be confirmed by clinical and molecular biology studies with larger sample sizes in the future.

## Figures and Tables

**Figure 1:** Comparison of curative effect between two groups of patients.

**Figure 2:** Comparison of ovulation rate and pregnancy rate between two groups.

**Table 1:** comparison of follicular size and endometrial thickness before and after intervention$[\bar{x}$±s].

Group	N	Follicular size(cm^2^)		Endometrial thickness(cm)	
		Before intervention	After intervention	Before intervention	After intervention
C group	50	1.22 ± 0.23	1.34 ± 0.28^a^	0.71 ± 0.14	0.88 ± 0.20^a^
R group	50	1.18 ± 0.16	1.51 ± 0.23^b^	0.77 ± 0.17	0.99 ± 0.23^b^
*t*		1.010	3.317	1.926	2.552
*P*		0.315	0.001	0.057	0.012

Note: the control group before and after intervention, aP<0.05; the study group before and after intervention, bP<0.05.

**Table 2:** comparison of ovulation between the two groups before and after intervention$[\bar{x}$±s，individual].

Group	N	Number of mature follicles		Ovulation number	
		Before intervention	After intervention	Before intervention	After intervention
C group	50	1.63 ± 0.36	2.45 ± 0.86^a^	1.50 ± 0.54	2.82 ± 0.84^a^
R group	50	1.60 ± 0.35	4.76 ± 0.90^b^	1.47 ± 0.56	4.48 ± 0.73^b^
*t*		0.422	13.122	0.273	10.547
*P*		0.674	0.001	0.786	0.001

Note: the control group before and after intervention, a P <0.05; the study group before and after intervention, b P <0.05.

**Table 3:** comparison of sex hormone levels between the two groups before and after intervention$(\bar{x}$±s，n =50).

Group	LH(IU/L)		FSH(IU/L)		T(nmol/L)		E_2_(pg/ml)	
	Before intervention	After intervention	Before intervention	After intervention	Before intervention	After intervention	Before intervention	After intervention
C group	12.57 ± 3.81	8.92 ± 2.33^a^	6.03 ± 1.21	5.47 ± 1.35^a^	6.72 ± 2.04	3.16 ± 0.91^a^	131.62 ± 20.62	119.33 ± 11.24^a^
R group	12.86 ± 3.45	6.13 ± 1.18^b^	5.90 ± 1.18	3.78 ± 1.06^b^	6.92 ± 1.83	1.95 ± 0.63^b^	132.07 ± 20.57	103.47 ± 12.08^b^
T value	0.385	7.554	0.418	6.962	0.516	7.730	0.109	6.797
*P* value	0.700	≤0.001	0.677	≤0.001	0.607	≤0.001	0.913	≤0.001

Note: the control group before and after intervention, a P <0.05; the study group before and after intervention, b P <0.05.

**Table 4:** comparison of menstrual score and serum CTRP3 and CTRP15 levels before and after intervention(^−^x ± s， n =50).

Group	Menstruation score (score)		CTRP3(IU/L)		CTRP15(nmol/L)	
	Before intervention	After intervention	Before intervention	After intervention	Before intervention	After intervention
C group	6.41 ± 2.14	3.78 ± 1.68^a^	16.42 ± 3.33	11.42 ± 2.27^a^	13.57 ± 3.14	9.12 ± 1.85^a^
R group	6.50 ± 2.09	2.31 ± 1.28^b^	16.30 ± 3.28	9.41 ± 2.01^b^	13.49 ± 3.17	6.51 ± 1.20^b^
t value	0.213	4.921	0.182	4.688	0.127	8.369
*P* value	0.832	≤0.001	0.856	≤0.001	0.899	≤0.001

Note: the control group before and after intervention, aP<0.05; the study group before and after intervention, bP<0.05.

## Data Availability

No data were used to support this study.
